The article "Whole Exome Sequencing Facilitated the Identification of a Mosaic Small Supernumerary Marker Chromosome (sSMC)" was published in 2021. Journal: Biomed Res Int.

# Whole Exome Sequencing Facilitated the Identification of a Mosaic Small Supernumerary Marker Chromosome (sSMC)

**DOI:** 10.1155/2021/6258527

**Published:** 2021-07-02

**Authors:** Huan-xia Xing, Peng-bin Li, Li-min Cui, Jian-ye Jiang, Ning-ning Hu, Xiao-bin Zhang

**Affiliations:** ^1^Prenatal Diagnosis Center, Langfang Maternal and Child Health Care Hospital, Langfang, Hebei 065000, China; ^2^Department of Orthopaedics, Langfang Traditional Chinese Medicine Hospital, Langfang, Hebei 065000, China

## Abstract

Small supernumerary marker chromosomes (sSMCs) are a group of rare chromosomal anomalies, which pose challenges in the clinical practice of prenatal diagnosis and genetic counseling. This study enrolled an extended family with an underage male patient displaying infantile seizures, intellectual disability, and retarded speech and psychomotor function. A series of multiplatform genetic detections was conducted to explore the diagnostic variation. Whole exome sequencing (WES) and chromosomal microarray analysis (CMA) indicated a mosaic sSMC derived from the pericentromeric region of chromosome 8 in the patient, which was confirmed using cytogenetic methods. The proband and his mother, who carried this mosaic variant, exhibited strong phenotypic variability. We also ruled out the pathogenicity of a *KDM5C* variant by extended validation. Our results emphasized the capacity of WES to detect mosaic SMCs and the importance of mosaic ratios in the appearance and severity of symptomatic phenotypes.

## 1. Introduction

Small supernumerary marker chromosomes (sSMCs) are a group of rare chromosomal anomalies involving both numerical and structural variations with a size equal to or smaller than chromosome 20 in the same metaphase spread [1]. The incidence of sSMC ranges from 5/10000 to 1/5000 in newborns [2]. The sSMC can be derived from each of the 24 human chromosomes, may consist of continuous stretches of DNA from one or more chromosomes, may also be constituted from discontinuous parts of the same or different chromosomes, and contain hetero-and/or euchromatic DNA [3]. The sSMCs are preferentially detected in patients with either of three clinical conditions: (a) infertility, (b) physical and/or mental impairment, and (c) prenatally, in children with/without sonographic abnormalities [4–6]. Mosaicism is a frequent occurrence in sSMC cases and has been recently reported to be associated with sSMC from specific chromosomal derivations [1, 3].

In conventional clinical practice, sSMCs have always posed a challenge for prenatal diagnosis and genetic counseling [7]. Historically, the inadequacy of detection methods led to difficulties in the identification of sSMC, which has recently been overcome by the rapid development of molecular cytogenetic techniques. More attention is now being paid to understanding the correlation between genotype and phenotype associated with sSMCs, which is a difficult issue in mosaic cases [8, 9].

In this study, a family with an underage proband exhibiting severe intellectual disability and hypoevolutism was enrolled and submitted to a series of prospective molecular cytogenetic detection. A causative hereditary mosaic sSMC derived from chromosome 8 was identified, although the proband and his mother carrying it showed strong phenotypic variation. After the confirmation of this variant using multiplatform techniques and eliminating the interference of another sequence variant, we made the final etiological determination. The findings of this study further emphasized the uncertainty of clinical outcomes of mosaic sSMCs.

## 2. Material and Methods

### 2.1. Subjects

A family with a 5-year-old male patient was referred to our center. The patient was born to nonconsanguineous healthy parents with normal growth parameters after a full-term pregnancy. The mother was 38-year-old at delivery. At 2 days of age, he exhibited paroxysmal convulsions and was diagnosed with infantile seizures, acute bronchitis, myocardial injury, hepatic failure, anemia, and eczema at another institution. At the age of three months, he was admitted to another hospital for recurrent convulsions, where he was diagnosed with infantile spasms, psychomotor retardation, and upper respiratory tract infections. In our center, we further diagnosed him with intellectual disability, speech retardation, and muscular dystonia at 2-years-old, and subsequently conducted a comprehensive genetic analysis on the patient and members of his extended family.

### 2.2. Sample Collection and DNA Extraction

Peripheral blood samples were collected with written informed consent obtained from all participants. Genomic DNA was extracted using a QIAamp DNA Blood Mini Kit (Qiagen GmBH, Hilden, Germany), according to the manufacturer's instructions.

### 2.3. Whole Exome Sequencing (WES)

Trio WES was conducted on the proband and his parents. Briefly, the target-region sequences were enriched using the Agilent Sure Select Human Exon Sequence Capture Kit (Agilent, USA). The DNA libraries were then tested for enrichment by quantitative PCR, of which the size, distribution, and concentration were determined using an Agilent Bioanalyzer 2100 (Agilent, USA). The NovaSeq6000 platform (Illumina, Inc.), along with ~150 bp pair-end reads, was used to sequence DNA at a concentration of ~300 pM per sample using the NovaSeq Reagent kit. Sequencing raw reads (quality level *Q*30% > 90%) were aligned to the human reference genome (accession no. hg19/GRCh37) using the Burrows-Wheeler Aligner tool [10], and the PCR duplicates were removed using Picard (version 1.57). Variant calling was performed with the Verita Trekker® Variants Detection system (version 2.0; Berry Genomics, China) and the Genome Analysis Tool Kit (https://software.broadinstitute.org/gatk/). Then, the variants were annotated and interpreted using ANNOVAR (version 2.0) [11] and Enliven® Variants Annotation Interpretation systems (Berry Genomics), based on the common guidelines by the American College of Medical Genetics and Genomics (ACMG) [12]. To assist in the interpretation of pathogenicity, we referred to three frequency databases (1000G_2015aug_eas, https://www.internationalgenome.org; ExAC_EAS, http://exac.broadinstitute.org; gnomAD_exome_EAS, http://gnomad.broadinstitute.org) and HGMD Pro (version 2019) (Human Gene Mutation Database). Sanger sequencing using 3500DX Genetic Analyzer (Applied Biosystems, USA) was performed to confirm the variants.

### 2.4. Chromosomal Microarray Analysis (CMA)

CytoScan 750K (Affymetrix, USA) microarray was used to test for copy number variations (CNV), loss of homozygosity (LOH), uniparental disomy (UPD), and mosaicism, according to the manufacturer's instructions. The Affymetrix Gene Chip Command Console software (version 4.0) and Chromosome Analysis Suite (version 2.1) (Affymetrix, USA) were used to analyze the raw data.

### 2.5. Chromosomal Karyotyping

G-banding technology was performed to identify the chromosomal abnormalities according to the AGT cytogenetics laboratory manual [13]. The standard experimental procedure involved the PHA and colchicine-stimulated lymphocyte cultures, preparation of chromosome specimens, digestion by trypsin, G-band staining, and karyotype analysis, according to the ISCN-2016 [14].

### 2.6. Fluorescence In Situ Hybridization (FISH)

Fluorescence *in situ* hybridization (FISH) using the CEP8 probe was conducted to determine the proportion of mosaic sSMC.

## 3. Results

### 3.1. Identification of the Mosaic sSMC

The results of WES indicated an increase in genetic material around the pericentromeric segment of chromosome 8 in the patient sample (Figure 1; top row, red block), which was consistent with the results of CMA (Figure 2; second row, red block). Specifically, it was a segment spanning ~13.7 Mb in the 8p11.23q11.21 (8: 36919180_50674599 bp) of chromosome 8 (Figure 2(a)). Besides, CMA indicated that the mosaic ratio of this segment was ~20% in the proband. Further validation by karyotyping revealed that ~11% (11/100) of the metaphases of the proband contained an sSMC (Figure 2(b)). FISH with a CEP8 probe indicated that ~13% of the interphases had three signals, whereas the rest had two (Figures 2(c) and 2(d)).

The results of the WES of the parents revealed no significant CNVs (Figure 1; 2 rows below). Similarly, the CMA results showed “no variation with clinical significance” in both of the parents (data not shown). Later, 100 metaphase cells from each of the parents were analyzed, but no sSMC was identified (Figures 2(e) and 2(h)). However, FISH identified three interphases containing three signals of the CEP8 probe out of 100 cells from the mother's sample, whereas the father's cells showed none (Figures 2(g) and 2(j)). FISH on metaphases from both parents showed no extra signal either (Figures 2(f) and 2(i)). Therefore, the mosaic ratio of this sSMC in the mother was probably no more than 3%.

### 3.2. Exclusion of Interference from a Sequence Variant

From the patient, WES also screened out a questionable hemizygous missense variant with unknown clinical significance, namely, *KDM*5*C* : NM_004187 : c.1169G > A (p.R390Q) (Figure 3(a)). It was demonstrated that the amino acid residue (R390) affected by it remained conserved among species (Figure 3(b)). Subsequent validation with Sanger sequencing revealed that it was inherited from the heterozygous mother. Further analysis of the extended family indicated that other asymptomatic members also carried this variant (Figure 3(c)), meaning it did not coseparate with the disease.

## 4. Discussion

Since the use of only G-banding has little potential in the identification of sSMCs, it has always been a challenge in the regular cytogenetic analysis, especially prenatal [1]. Liehr and Weise reviewed 132 studies and demonstrated that sSMCs presented with a higher frequency in cases with antenatal ultrasonic abnormalities, hypoevolutism, and infertility (especially males) [6]. *De novo* sSMCs, particularly those combined with uniparental disomy (UPD), were assumed to be derived from incomplete trisomy rescue and often tended to form mosaics [15, 16], which corresponded to the increased maternal age reported in most *de novo* cases [17, 18]. Moreover, chromothripsis explains why some sSMCs are formed by noncontiguous regions of a given chromosome [16].

In this study, a hereditary mosaic sSMC derived from the pericentromeric region of chromosome 8 was identified. Both the proband and his mother carried this sSMC, although at different mosaic rates. According to the results of multiplatform testing, although the proportion of mosaicism in the blood sample did not necessarily match that in other tissues, it could only be roughly represented [3]; yet, the proportion of the proband was considerably higher than that of his asymptomatic mother. According to the literature, the mosaic pericentromeric sSMC(8), or r(8), is a recurrent anomaly that has been often reported, although involving fragments with different sizes and numbers of genes in various cases. It was demonstrated that patients carrying this variation exhibited a wide spectrum of symptoms, ranging from completely normal to severe developmental delay, mental abnormities, infertility, and dysmorphic facies (Table 1). We infer that several factors may be associated with phenotypic severity, such as (a) specific genes contained in redundant sSMC, (b) the presence of UPD, and (c) mosaic ratio in pivotal organs and tissues. In this study, since the results of CMA suggested the absence of a UPD situation, it is presumed that the repetition of some crucial genes in this segment caused the phenotypes. The detected segment contained 54 OMIM genes (https://www.deciphergenomics.org/; location chr8: 36919180_50674599), of which *KAT6A* (MIM ∗601408) was associated with mental retardation (autosomal dominant 32) characterized by microcephaly and psychomotor developmental delay, while *SLC20A2* (MIM ∗158378) was associated with the calcification of basal ganglia (idiopathic 1) characterized by a wide spectrum of neuropsychiatric symptoms (https://www.omim.org/). We proposed that these genes may play a pivotal role in disease development. However, further research is needed to determine the exact etiology for this patient. Moreover, based on the results of FISH, the mosaic ratios in both the mother and the patient were slightly varied at a low level, although this led to a strong intrafamily phenotypic variability. This phenomenon is unique and deserves further study. Besides, since we did not see the sSMC in the mother's metaphase, we cannot rule out the probability that the mother carries a mosaic trisomy-8 karyotype. If that were the case, the proband's sSMC would be the result of partial trisomy rescue [15]. Future pregnancies of the couple are still at high risk, and prenatal diagnosis is recommended.

The suspicious nonsynonymous hemizygous missense variant carried by the proband *KDM*5*C* : NM_004187 : c.1169G > A was also given enough attention, as the *KDM5C* gene (MIM ∗314690) is associated with X-linked mental retardation (syndromic, ClaesJensen type, MIM #300534) characterized by severe mental retardation, slowly progressive spastic paraplegia, facial hypotonia, and maxillary hypoplasia. Further validation of the pedigree revealed that the variant did not coexist with the disease phenotype throughout the extended family, suggesting that it might not be causative. However, the actual effect of this variant on gene function also requires the finalization of deep functional experiments, as there may also be the involvement of incomplete penetrance and phenotypic variability in it.

Advances in molecular genetics over the past 15 years have made it possible to determine the size of sSMCs and the specific genes contained therein [9, 19, 20]. The results of WES in this study may also suggest the existence of sSMC, even mosaic, which highlights that WES or WGS (whole genome sequencing) is an intensive method that can detect sequence variation, copy number variation, and structural variation simultaneously. However, multiplatform experimental testing, especially using traditional cytogenetic methods such as karyotyping and FISH, remains indispensable, especially for prenatal cases.

In conclusion, we present a novel mosaic sSMC containing the 8p11.23q11.21 segment identified using multiplatform techniques, which was associated with infantile seizures, intellectual, and motor retardation. Our results highlight the ability of WES to detect mosaic sSMCs apart from sequence variation, emphasizing the importance of mosaic ratios in determining the appearance and severity of symptomatic phenotypes.

## Figures and Tables

**Figure 1:** Molecular indications of the sSMC in the proband. (Top two rows: WES result of the proband, extra materials demonstrated in the red block; second row: CMA result of the proband with CytoScan 750K, extra materials demonstrated in the red block; four rows below: WES results of the parents).

**Figure 2:** Cytogenetics of the family. (a) Detailed CMA result of the proband. (b) Metaphase of the proband by G-banding (red arrow indicates the sSMC). (c) The interphase nucleus of the proband with three signals of the CEP8 probe. (d) The interphase nucleus of the proband with two signals of the CEP8 probe. (e) Metaphase of the proband's mother. (f) FISH on metaphase of the mother with two signals of CEP8. (g) FISH on interphase of the mother with three signals of CEP8. (h) Metaphase of the proband's father. (i) FISH on metaphase of the father with two signals of CEP8. (j) FISH on interphase of the father with two signals of CEP8.

**Figure 3:** Family validation of the *KDM*5*C* : c.1169G > A variant. (a) WES data indicated that the proband was hemizygous with this variant (top row), the father was wild-type (midrow), and the mother was heterozygous (bottom row). (b) The affected amino acid (R390) remains conserved across several species. (c) The status of this variant across the family.

**Table 1:** Pericentromeric sSMC(8) reported in related literature.

Authors; year	PMID∗	Size (range) of sSMC	Number of carriers	Mosaic ratio (%)∗	Detection methods∗	Clinical manifestations∗
Shao et al.; 2020	32127158	~45.2 Mb (8p12_q21.13; 36,013,636e81,263,140 bp)	1	60 (karyotyping); 51 (SNP array)	Karyotyping; SNP array	Congenital hypoplasia of the tongue; birth history of abnormal child
Chen et al.; 2016	28040133	~11 Mb (8p11.22_q11.21; 39,136,065–49,725,726 bp)	1	55 (karyotyping); 70–80 (aCGH); 44 (FISH)	FISH; aCGH;	Obesity, intellectual disability, attention deficit hyperactivity
Ahram et al.; 2016	27980747	~11 Mb (8p11.22_q11.21; 38,989,813–50,283,147 bp)	1	60 (karyotyping)	SNP array; QF-PCR	Fetal pyelectasis; autism spectrum, hypermetropia; maternal UPD
Chen et al.; 2012	23040926	~43 Mb (8p22_q12.1; 18,100,180–61,104,884 bp)	1	20 (amniocytes karyotyping)	FISH; aCGH; QF-PCR	Fetal pyelectasis; normal after birth
Chen et al.; 2010	21199754	~4.4 Mb (8p11.21_q11.1; 42,637,263–47,062,180 bp)	1	93	Karyotyping; FISH; aCGH; MLPA	Left multicystic kidney, mild ventriculomegaly (perinatal)
Bettio et al.; 2008	18076101	~5 Mb (8p11.21_q11.21)	1	50 (chorionic villi); 89 (amniocyte); 96 (lymphocytes)	aCGH; FISH; karyotyping	Intellectual delay
Weimer et al.; 2006	16470789	/(8p11.1_q11.1)	1	73^#^ (48,XX,+mar1,+mar2[68]/47,XX,+mar1[19]/47,XX,+mar2[6]/46,XX [8])	Karyotyping; FISH	Cooccurrence of a partial Y-chromosome; Klinefelter syndrome signs, mild facial anomalies, and severe speech delay
Gole and Biswas; 2005	15662692	/(8p11.2_q11.2)	1	50	Karyotyping; FISH	Normal after birth
Herry et al.; 2004	15211653	/(8p11_q11)	1	76 (case 1)	Karyotyping; FISH	Case 1: mild intellectual delay, spontaneous miscarriage
Loeffler et al.; 2003	12503109	/(8p12_q12)	1	70	Karyotyping; FISH	Muellerian aplasia, renal and skeletal anomalies, minor mental, genital and facial anomalies.
Daniel and Malafiej; 2003	12599184	/(/)	3	34 (case 1); 27 (case 2); 54 (case 3)	Karyotyping; FISH; microsatellite analysis	Case 1: infertile, IQ 80–85, central obesity; case 2: normal; case 3: severe intellectual delay, mild ataxia, dysmorphic facies
Starke et al.; 1999	10590438	/(8p11_q11)	1	70 (by banding); 54 (by FISH)	Karyotyping; FISH; microsatellite analysis	Slight pyelectasia, echogenic intestine (prenatal ultrasonography); normal development (9 months); no UPD
Rothenmund et al.; 1997	9332666	/(/)	3	98 (1st D); 97 (2nd D); 10 (F)	Q-banding; FISH	1st D: developmental delay, autistic behaviors; 2nd D: cardiac anomalies; F: normal
Blennow et al.; 1993	8328459	/(/)	1	40 (amniocytes); 72 (fibroblasts)	Q-banding; FISH	Motor retardation, hypertelorism, bulbous nose, low-set ears, pes equinovarus, narrow shoulders, and an external nipple

∗PMID: PubMed ID (https://pubmed.ncbi.nlm.nih.gov/); D: daughter; F: father; FISH: fluorescence in situ hybridization; aCGH: array comparative genomic hybridization; MLPA: multiplex ligation-dependent probe amplification; QF-PCR: quantitative fluorescent polymerase chain reaction; SNP: single nucleotide polymorphism; UPD: uniparental disomy. # mar2 represents the sSMC(8).

## Data Availability

The underlying data supporting the results of this study can be required to the corresponding author based on reasonable demand.
